# Parthenolide Augments the Chemosensitivity of Non-small-Cell Lung Cancer to Cisplatin *via* the PI3K/AKT Signaling Pathway

**DOI:** 10.3389/fcell.2020.610097

**Published:** 2021-02-05

**Authors:** Li-Mei Wu, Xiao-Zhong Liao, Yan Zhang, Zi-Rui He, Shi-Qing Nie, Bin Ke, Lin Shi, Jian-Fu Zhao, Wen-Hui Chen

**Affiliations:** ^1^Department of Oncology, The First Affiliated Hospital of Jinan University, Guangzhou, China; ^2^Department of Oncology, The First Affiliated Hospital of Guangzhou University of Chinese Medicine, Guangzhou, China; ^3^Department of Traditional Chinese Medicine, Cancer Center of Sun Yat-sen University, Guangzhou, China; ^4^Department of Traditional Chinese Medicine, Zhujiang Hospital, Southern Medical University, Guangzhou, China

**Keywords:** PTL, DDP, combination, synergistic effect, NSCLC, PI3K/Akt pathway

## Abstract

The mortality rate of non-small-cell lung cancer (NSCLC) remains high worldwide. Although cisplatin-based chemotherapy may greatly enhance patient prognosis, chemotherapy resistance remains an obstacle to curing patients with NSCLC. Therefore, overcoming drug resistance is the main route to successful treatment, and combinatorial strategies may have considerable clinical value in this effort. In this study, we observed that both parthenolide (PTL) and cisplatin (DDP) inhibited the growth of NSCLC cells in a dose- and time-dependent manner. The combination of PTL and DDP presented a synergistic inhibitory effect on NSCLC at a ratio of 50:1. The combination of PTL and DDP synergistically inhibited cell migration and invasion, inhibited cell cycle progression, and induced apoptosis of A549 and PC9 cells. Bioinformatics and network pharmacology analysis indicated that PTL may primarily affect the phosphatidylinositol 3-kinase (PI3K)-AKT signaling pathway. After treatment with PTL and DDP either alone or in combination, Western blot analysis revealed that the proteins levels of Bax and cleaved Caspase-3 were upregulated, while p-PI3K, p-Akt, Caspase-3, and Bcl-2 proteins were downregulated. Among these alterations, the combination of PTL and DDP was found to exhibit the most significant effects. PTL might therefore be considered as a new option for combination therapy of NSCLC.

## Introduction

Lung cancer is the most common and most aggressive malignancy, as well as the principal cause of cancer-related deaths in both men and women all over the world (Siegel et al., 2018) and in China (Chen et al., 2016). About 80–85% patients with lung cancer are diagnosed with non-small cell lung cancer (NSCLC) (Chen et al., 2016; Siegel et al., 2018). In recent decades, important progress has been made in the diagnosis and treatment strategies of NSCLC, although there has been no significant improvement in its prognosis, and the 5-year overall survival rate is still <15% (Chen et al., 2014). Platinum-based chemotherapy is still the standard-of-care for most patients who suffer from advanced NSCLC (Rossi and Di Maio, 2016). Nevertheless, toxicity, drug resistance, and high risk of death are seen clinically, underlining that the medication strategies require to be optimization. There are two types of drug resistance: primary resistance which appertains to chemoresistance prior to chemotherapy, and acquired resistance which emerges following chemotherapy (Kelland, 2007). The common mechanisms of drug resistance mainly include increased drug efflux from cancer cells, reduced uptake of drugs, modification of oncogenes, and inhibition of drug-induced apoptosis (Hamilton and Rath, 2014). Ultimately, the resistance leads to chemotherapy failure and therefore a poor prognosis.

DDP, also known as cisplatinum or cis-diamminedichloroplatinum (II), is a chemotherapeutic drug (Dasari and Tchounwou, 2014). It has been used to treat a variety of solid malignancies, including testicular, ovarian, head and neck, colorectal, bladder, and lung cancers (Gridelli et al., 2015). Cisplatin exerts anticancer effects through multiple mechanisms, but its utmost (and best understood) mode of action involves the generation of DNA lesions followed by the activation of DNA damage response and the induction of mitochondrial apoptosis (Dasari and Tchounwou, 2014). Cisplatin treatment often induces the development of chemoresistance, leading to therapeutic failure and plentiful unfavorable side effects such as serious kidney problems, allergic reactions, declining immunity to infections, gastrointestinal diseases, hemorrhage, as well as hearing loss found particularly in young patients (Dasari and Tchounwou, 2014). Because cisplatin is the main therapeutic option in some clinical settings, the development of chemosensitization strategies has become a clinically significant goal. In addition, combination therapies with cisplatin and other drugs have been taken into high consideration to surmount drug-resistance and lessen toxicity.

Fortunately, natural products with various chemical structures and pharmacological effects can serve as effective drug-resistant substances (Thomford et al., 2018). PTL, originally isolated from *Tanacetum parthenium* L., is a prominent and naturally occurring germacranolide, which has shown cytotoxicity in multifarious human cancer cells but not in normal cells (Ghantous et al., 2013). PTL has been found to have anti-inflammatory (Wang et al., 2016), antioxidant (Farzadfar et al., 2016), and antitumor activity in a variety of cancers, including breast (Araujo et al., 2019), acute myeloid leukemia (Darwish et al., 2019), and non-small cell lung cancer (Zhang et al., 2009).

Despite the anticancer effect of PTL reported previously in several cancer cell lines, the effect of co-treatment with PTL and DDP for synergistic inhibition of NSCLC cells has not been well-explored. The aim of this study was to investigate the potential synergistical effects of the combination of PTL and DDP on NSCLC as well as the related mechanism.

## Materials and Methods

### Reagents, Cell Lines, and Cell Culture

Parthenolide and cisplatin (Figure 1) were obtained from Santa Cruz Biotechnology (Dallas, USA). A549, PC9, H1299, and BEAS-2B cell lines were generously provided by the State Key Laboratory of Oncology in South China. They were cultivated in RPMI 1640 medium supplemented with 10% fetal bovine serum, L-glutamine, gentamycin, and penicillin/streptomycin, and cultured at 37°C in a humidified atmosphere containing 5% CO_2_.

**Figure 1:** 2D structure of DDP **(A)** and PTL **(B)** (obtained from PubChem compound, http://pubchem.ncbi.nlm.nih.gov/).

### Cell Viability Assay

Cell viability was evaluated using a Cell Counting Kit-8 (CCK8) assay. Exponentially growing cells were inoculated in 96-well culture plates (~6,000 cells/well in 100 μL medium), cultivated overnight, and incubated with a series of concentrations of PTL (0–100 μM) or DDP (0–2 μM) for 48 h. Then 10 μL of CCK8 solution was added to each well, the plate was incubated at 37°C for 2 h, and the absorbance (A) was measured at 450 nm on a microplate plate reader (Thermo Scientific, Rockford, IL, USA). The inhibition rate was calculated as follows: (A control - A treated)/A control × 100%, where A treated and A control are the absorbance of the treated and control cells, respectively.

### Calculation of the Combination Effect Index

The inhibitory effects of PTL and DDP were confirmed by CCK8 assay. We employed the combination index (Cl) depicted by Chou and Talalay for analysis and carried out the analysis by utilizing the CalcuSyn software. CI < 1 denotes synergism; CI = 1 denotes summation; and CI > 1 denotes antagonism.

### Wound Healing Assay

A549 and PC9 cells were plated into 6-well plates (1 × 10^6^ mL/well). When the cell density was about 90% after 24 h, serum-free medium was used to starve the cells for 24 h. Confluent monolayer cells were scratched in a straight line using a 100 μL pipette tip. The exfoliated cells were cleared with PBS (GIBCO) wash three times. Then the serum free RPMI1640 containing various drugs was used to culture the cells and the cells are allowed to heal the wounds for 48 h. At the same place where cells were scratched, pictures (magnification, 10×) were taken at 0 and 24 h. Ultimately the Adobe Photoshop CS6 software was used to determine the migration length of cells according to the change of wound size.

### Transwell Invasion Assay

A549 and PC9 cells were incubated in serum-free RPMI1640 for 24 h. Subsequently, cells (6 × 104) in 600 μL serum-free medium containing various drugs were plated on the top compartment of transwell filters, which were covered by thin layers of matrigel basement membrane matrix, with 700 μL medium containing 10% FBS in the bottom compartment. The transwell filters were cultured at 37°C with 5% CO_2_ for 48 h. After that, the cells adhering to the bottom membrane were fixated in 4% paraformaldehyde for 30 min, and subsequently dyed with 0.5% CV solution for 15 min at room temperature. Ultimately, the transwell filters were inverted and observed under a microscope (magnification, 100×) for photographic recording and the number of cells on the bottom surface was counted. Five random fields were counted per filter in all groups.

### Cell Colony Formation Assay

Cells were trypsinized single cells were obtained and seeded in 6-well plates at a density of 500 cells/well. After 10 days of culture, colonies were fixed with methyl alcohol and stained with crystal violet, and the colony formation ratio was calculated.

### Cell Cycle Distribution Analysis

A Cell Cycle Detection Kit obtained from 4A Biotech Co., Ltd. (Beijing, China) was employed to detect the cell cycle distribution. Briefly, A549 and PC9 cells were inoculated in six-well plates (1 × 10^6^ cells/well) and cultured overnight, and then cells were incubated with PTL or DDP alone or in combination for 48 h. After that, cells were rinsed with cold phosphate-buffered saline (PBS) and immobilized with 70% ethyl alcohol overnight. After washes with PBS, cells were stained with propidium iodide (10 μg/mL) in the presence of RNase (1 g/L), 1 g/L sodium citrate, and 0.5% Triton X-100 (v/v) in the dark for 30 min. Then cells were collected for cell cycle distribution analysis using an ACEC NovoCyte flow cytometer equipped with Novoexpress (Becton Dickinson, San Jose, CA, USA).

### Cell Apoptosis Analysis

An Annexin V-FITC apoptosis detection kit obtained from 4A Biotech Co., Ltd. (Beijing, China) was used to detect cell apoptosis. A549 and PC9 cells were seeded in six-well plates and cultured overnight. After exposure to PTL or DDP alone or in combination for 48 h, the cells were harvested, resuspended in 500 μL of incubation buffer containing Annexin V-FITC and PI, and incubated for 30 min in the dark. The cells were then washed and subjected to apoptosis analysis using an ACEC NovoCyte flow cytometer furnished with Novoexpress.

### Xenograft Tumor Assay in Nude Mice

Nude female BALB/c-nu/nu mice (4–6 weeks) were obtained from the Institute of Laboratory Animal Sciences, Chinese Academy of Medical Sciences, Beijing, China, and placed in a specific pathogen-free (SPF) environment. A549 cells (3 × 10^6^) in 0.2 mL of PBS were inoculated into the flanks of the mice. When tumors became palpable, mice were subdivided into four groups of six. **Figure 7A** shows the *in vivo* treatment regimen with a variety of concentrations of PTL or DDP. PTL and vehicle control were administrated daily *via* intraperitoneal (I. P.) injection, while DDP was administrated every 5 days *via* I. P. injection. The tumor volumes were measured at the beginning of the treatment and every 4 days during treatment by measuring the length (L) and width (W) of the tumors. The tumor volume was calculated by the following formula: *v* = length × (width)^2^/2. Tumors were excised and weighed on the second day after the last injection. All experiments were approved by the Institutional Animal Care and Use Committee of Sun Yat-sen University and performed in accordance with national ethical guidelines.

### Potential Target Identification Based on Pharmmapper

PharmMapper (http://lilab.ecust.edu.cn/pharmmapper/index.php) consists of a huge internal repertoire of a pharmacophore database, which is pulled out from all the targets in TargetBank, DrugBank, BindingDB, and PDTD. PharmMapper stores and accesses over 7,000 receptor-based pharmacophore models (information about 1,627 drug targets can be found, and 459 of which are human protein targets). First, the SDF format of PTL was downloaded from PubChem Compound (https://www.ncbi.nlm.nih.gov/pccompound/) and then uploaded to PharmMapper. After exactly setting the parameters, target recognition was performed, and the information relating to the first 300 potential protein targets was acquired.

### Bioinformatics and Network Pharmacology Analysis

Based on the DAVID database (https://david.ncifcrf.gov/), we imported the top 300 potential targets, selected Homo sapiens, and then carried out Gene Ontology (GO) analysis and Kyoto Encyclopedia of Genes and Genomes (KEGG) pathway enrichment analysis. The information associated with the first 100 potential pathways was acquired. A parameter enrichment gene count ≥2 and hypergeometric analysis were used for testing significance threshold with a *P* < 0.05. For a KDR value <0.05 (Q), we selected the Top 20 pathway, and mapped senior bubbles by the OmicShare website (http://www.omicshare.com/).

### Western Blot Analysis

Cells were harvested and processed in RIPA lysis buffer supplemented with 1% phenylmethanesulfonyl fluoride and 1% phosphatase inhibitor. The soluble protein fractions were extracted after centrifugation at 1.35 × 10^4^ g for 10 min. The protein concentrations were tested using a BCA kit. Around 30 mg of proteins were separated by 8–12% sodium dodecyl sulfate-polyacrylamide gel electrophoresis (SDS-PAGE), transferred to PVDF membranes, and incubated with different primary antibodies overnight at 4°C. Membranes were then washed and incubated with proper secondary antibodies. Signals were detected using an ECL chemiluminescence detection kit.

### Statistical Analysis

SPSS 24.0 software (IBM, NY) was employed to performed statistical analysis. Statistical comparisons were performed through independent samples *t*-test or one-way analysis of variance (ANOVA). Data measurements are indicated as mean values ± standard deviation. The value of *p* < 0.01 was considered statistically significant.

## Results

### Co-treatment With PTL and DDP Concurrently Inhibited the Proliferation of NSCLC Cells

It was observed that both PTL and DDP inhibited the proliferation of NSCLC cells in a dose-dependent manner. After 48 h treatment with PTL, the IC_50_ values were 29.423, 23.21, 47.70, and 119.67 μM for A549, PC9, H1299, and BEAS-2B cell lines, respectively. Similarly, the IC_50_ values obtained after DDP treatment were 0.89, 0.73, 0.93, and 0.68 μM for A549, PC9, H1299, and BEAS-2B cell lines, respectively (Figure 2). We also treated the cell lines with a combination of PTL and DDP (the PTL:DDP molar ratio of 50:1) for 48 h. The results showed that, when compared with single drug therapy, the combination drug therapy had a stronger inhibitory effect on cell proliferation. The synergistic effects of drug combination therapy were observed in the A549, PC9, and H1299 cell lines with different Fa values, but not in the BEAS-2B cell line. Table 1 lists the summary of the CI and the concentrations of the individual drugs used in combination at 50% Fa.

**Figure 2:** Proliferative inhibitory effect of PTL, DDP, and the combination treatment on NSCLC cells. Drug concentration–cell viability curves were generated as the viable cell percentage based on the cell viability assay **(A,C,E,G)**. Synergistic effects between PTL and DDP are presented as Fa-CI plots **(B,D,F,H)**. Data are from three repeated experiments with quadruplicate wells (mean ± SD).

**Table 1:** Summary of CI value and the concentration of separate drugs in combination at 50% Fa.

**Drug combination**	**Fa = 0.5**			
	**A549**	**PC9**	**H1299**	**BEAS-2B**
DDP + PLT				
CI	0.69832	0.71184	0.74952	1.71719
DDP (μM)	0.38906	0.35321	0.48497	0.44289
PLT (μM)	9.72652	8.83035	12.1244	11.0722

### Cooperation of PTL and DDP Synergistically Suppressed the Migration and Invasion of NSCLC Cells

We used wound healing assay and transwell assay to evaluate the effects of individual PTL and DDP or combination of these two drugs on the migration and invasion of A549 and PC9 cells. Figure 3 shows that both the migration distances and invaded cell numbers were reduced markedly after 48 h treatment with either individual drugs or a combination of PTL and DDP. Furthermore, the combination treatment resulted in the smallest values for both migration distance and aggressive cell number, suggesting the combination of PTL and DDP exerted a more significant inhibition on cell migration and invasion than each of them alone.

**Figure 3:** PTL and DDP suppress the migration and invasion ability of A549 and PC9 cells. Representative images of wound healing and transwell assays **(A,B)** following 48 h of treatment with 30 μM PTL, 0.75 μM DDP alone, and 0.2 μM DDP and 10 μM PTL in combination. Histograms depict the average migrated distance **(C,E)** and the number of invasive cells **(D,F)**, respectively. All data are shown as the mean ± SD of three independent experiments. *P < 0.05, **P < 0.01 or ***P < 0.001 vs. the control group (magnification, × 100; scale bars, 100 μm).

### Co-treatment With PTL and DDP Coordinately Inhibited the Cell Colony Formation of NSCLC Cells

As showed in Figure 4, compared with untreated controls, PTL, DDP, and the combination of them all significantly inhibited cell colony formation of A549 and PC9 cells. Similarly, the combination of PTL and DDP exerted a more significant inhibition on cell colony formation than each of them alone.

**Figure 4:** Effect of PTL and DDP alone and in combination on cell clone formation. Representative images of clone formation in A549 **(A)** or PC9 cells **(C)** following 10 days of treatment with 30 μM PTL, 0.75 μM DDP alone, and 0.2 μM DDP and 10 μM PTL in combination. Histograms depict the average clone formation of A549 **(B)** and PC9 **(D)**. All data are shown as the mean ± SD of three independent experiments. ***P < 0.001 vs. the control group (magnification, × 100; scale bars, 100 μm).

### Co-treatment With PTL and DDP Synergistically Arrested the Cell Cycle of NSCLC Cells

After verifying the anti-proliferative effect of PTL and DDP, flow cytometry (FCM) was used to analyze the cell cycle of the treated NSCLC cells. As illustrated in Figure 5, PTL and DDP both arrested A549 and PC9 cells at S and G2 phases, while the combination of PTL and DDP showed a more significant effect in arresting PC9 cells at S and G2 phases.

**Figure 5:** Effect of PTL and DDP alone and in combination on cell cycle arrest. The percentage of cells in the G1, S, or G2 phase in A549 **(A)** or PC9 cells **(C)** treated with 30 μM PTL, 0.75 μM DDP alone, and 0.2 μM DDP and 10 μM PTL in combination for 48 h. Data represent the cell population in cell cycle arrest of A549 **(B)** and PC9 **(D)** cells. All data are shown as the mean ± SD of three independent experiments. *P < 0.05, **P < 0.01 vs. the control group.

### Co-treatment With PTL and DDP Synergistically Induced Apoptosis in NSCLC Cells

As shown in Figure 6, both the PTL and DDP individual drug treatments and the drug combination enhanced the ratio of early and late apoptosis in A549 and PC9 cells. Additionally, the combination of PTL and DDP was more efficient at inducing apoptosis compared to the single treatment (PTL + DDP vs. PTL, *p* = 0.0004; PTL + DDP vs. DDP, *p* = 0.0006).

**Figure 6:** Effect of PTL, DDP alone, and in combination on apoptosis. Representative profiles showing apoptosis in A549 **(A)** or PC9 cells **(C)** treated with 30 μM PTL, 0.75 μM DDP alone, and 0.2 μM DDP and 10 μM PTL in combination for 48 h. Data represent the cell population in cell cycle arrest of A549 **(B)** and PC9 **(D)** cells. All data are shown as the mean ± SD of three independent experiments. **P < 0.01, ***P < 0.001 vs. the control group.

### Co-treatment With PTL and DDP Synergistically Suppressed A549 Cell Xenograft Tumor Growth

Figure 7 shows the experimental setup of the *in vivo* animal experiment, including A549 cell seeding and drug treatment. Our next step was to study the effects of PTL and DDP on the growth of xenograft NSCLC tumors. It was found that the xenograft tumors in the control group grew faster than those in the group treated with the tested drugs. In addition, compared with PTL and DDP monotherapy, the combination of PTL and DDP had a more significant inhibitory effect on tumor growth (PTL + DDP vs. PTL, *p* = 0.004; PTL + DDP vs. DDP, *p* = 0.005). These results indicated that the anti-tumor effect of DDP *in vivo* could be effectively enhanced by PTL.

**Figure 7:** PTL combined with DDP inhibits NSCLC xenograft tumor growth. Time line of NSCLC cell inoculation and drug treatment **(A)**. Time courses of animal weight **(B)**. The tumor volume of all groups was measured every 4 days, beginning the first day after injection until the study end point **(C)**. Tumors derived from A549 cells in six male nude mice are presented **(D)**. The tumor weight of all groups was measured and compared, ***P < 0.001 vs. the control group **(E)**. Data are presented as mean ± SD. **P < 0.01 or ***P < 0.001. *N* = 5 in each group.

### Potential Target Proteins of PTL and the Bioinformatics and Network Pharmacology Analysis

The relevant information of the first 300 potential protein targets of PTL was obtained utilizing PharmMapper (Table 2). We conducted gene ontology (GO) analysis and Kyoto Encyclopedia of Genes and Genomes (KEGG) pathway enrichment analysis according to the DAVID database (https://david.ncifcrf.gov/). The obtained bioinformatics analysis was depicted in Figure 8, suggesting that PTL might play a role, mainly through affecting the PI3K/Akt signaling pathway.

**Table 2:** Potential targets of parthenolide by PharmMapper.

**Pharma model**	**Uniplot**	**Num feature**	**Fit**	**Norm fit**	***z*-score**
1reu	BMP2	3	2.975	0.9917	1.7192
2p3g	MAPK2	3	2.966	0.9888	1.75996
1j96	AK1C2	3	2.954	0.9848	1.89866
1w8l	PPIA	3	2.935	0.9783	1.64874
2oji	MK01	3	2.916	0.9719	1.42276
3dej	CASP3	3	2.723	0.9076	0.89396
3gam	NQO2	3	2.606	0.8686	0.64813
1xdd	ITAL	3	2.543	0.8478	0.09328
2vwu	EPHB4	3	2.465	0.8218	0.1209
1okl	CAH2	3	2.382	0.794	−0.3892
1n7i	PNMT	4	2.99	0.7474	1.73609
1mkp	DUS6	4	2.975	0.7437	1.5315
1x97	ALDR	3	2.202	0.7341	−0.4667
1fdu	HSD17B1	4	2.928	0.7319	1.38111
2h8h	SRC	4	2.927	0.7317	1.5454
2zas	ERR3	4	2.922	0.7304	1.27297
1m17	EGFR	4	2.891	0.7228	1.33827
2o65	PIM1	3	2.158	0.7194	−1.4526
1dic	CFAD	4	2.87	0.7176	1.3316
1vjy	TGFR1	4	2.848	0.712	1.1212
1sqn	PRGR	4	2.827	0.7068	1.05616
1j78	VTDB	4	2.789	0.6972	0.07214
2wi1	HSP90AA1	4	2.78	0.6951	0.96209
1dig	C1TC	4	2.761	0.6903	1.07111
1soj	PDE3B	4	2.758	0.6895	1.00205
1rkp	PDE5A	4	2.737	0.6842	0.91313
2ao6	ANDR	4	2.734	0.6834	0.69589
1e7a	ALBU	3	2.047	0.6824	−1.3033
2b1v	ESR1	4	2.729	0.6822	0.8369
3f7z	GSK3B	5	3.386	0.6772	3.03183
3f5p	IGF1R	4	2.677	0.6691	0.5812
1mkd	PDE4D	4	2.647	0.6617	0.43777
1mx1	EST1	4	2.633	0.6582	0.2642
2ywp	CHK1	4	2.604	0.6511	0.43158
2pe0	PDPK1	4	2.548	0.637	0.09329
1hak	ANXA5	4	2.482	0.6204	−0.8744
1b6a	AMPM2	4	2.481	0.6201	0.15918
1csb	CATB	4	2.443	0.6107	−0.2588
1shl	CASP7	4	2.416	0.6041	−0.3164
1p0p	CHLE	4	2.403	0.6008	−0.501
1d3g	PYRD	4	2.403	0.6007	−0.5732
1s1p	AK1C3	5	2.982	0.5964	1.44379
2abi	MCR	5	2.976	0.5953	1.42687
3czr	DHI1	5	2.97	0.5939	0.80992
1fzv	PLGF	5	2.958	0.5915	1.4615
1ov4	ST2A1	5	2.93	0.5859	0.36594
2zaz	MAPK14	5	2.915	0.5829	0.92383
1oiz	TTPA	5	2.912	0.5824	0.87911
1x70	DPP4	5	2.908	0.5817	1.12942
2c6i	CDK2	5	2.904	0.5808	0.91187
3fzk	HSPA8	4	2.321	0.5802	−0.5686
2rfn	MET	5	2.888	0.5776	1.08595
1xil	SOD2	5	2.877	0.5754	1.22561
1cg6	MTAP	5	2.852	0.5704	0.153
2f57	PAK7	5	2.851	0.5701	1.10983
3blr	CCNT1	5	2.841	0.5681	1.26335
1nwe	PTN1	5	2.828	0.5656	0.487
1mrq	AK1C1	5	2.82	0.5639	0.70797
2uvy	PRKACA	5	2.766	0.5531	0.90246
1pl6	DHSO	5	2.76	0.5521	0.19208
1yk7	CATK	5	2.751	0.5502	0.80829
1h6g	CTNA1	5	2.703	0.5405	0.41404
1m9j	NOS3	4	2.154	0.5384	−1.2797
2uzb	CCNA2	5	2.684	0.5369	0.29338
1dvu	TTHY	5	2.668	0.5336	−0.1348
2ok1	MK10	5	2.659	0.5318	0.45911
2byh	HS90A	5	2.656	0.5313	0.5925
1oec	FGFR2	5	2.638	0.5276	−0.0936
1d4p	THRB	5	2.596	0.5191	−0.648
1s95	PPP5	4	2.075	0.5188	−1.6801
1jj9	MMP8	5	2.588	0.5175	−0.087
1ctr	CALM	5	2.585	0.5171	−0.5541
1gse	GSTA1	6	3.041	0.5068	0.93213
1utt	MMP12	5	2.525	0.5051	−0.3739
1fm6	PPARG	4	2.006	0.5015	−2.3739
1dxo	NQO1	6	2.953	0.4921	0.94948
1fls	MMP13	6	2.947	0.4911	0.58991
1ro9	PDE4B	6	2.939	0.4898	0.84835
2fl6	KIF11	5	2.445	0.489	−0.6016
1kdk	SHBG	6	2.923	0.4871	0.83623
2p3t	FA10	6	2.906	0.4844	0.96818
1sm2	ITK	6	2.903	0.4839	0.49905
1xvp	NR1I3	6	2.899	0.4832	0.6173
1lrm	PH4H	5	2.404	0.4808	−0.1287
1r7t	BGAT	6	2.872	0.4787	0.932
2fv5	ADA17	6	2.863	0.4771	0.69919
1qab	RET4	6	2.837	0.4728	0.40275
1ju6	TYSY	6	2.822	0.4703	0.77136
2i6b	ADK	6	2.765	0.4608	−0.1426
1hy7	MMP3	6	2.763	0.4604	−0.1544
1i7g	PPARA	6	2.747	0.4579	0.15588
11gs	GSTP1	7	3.186	0.4551	0.95262
1q22	ST2B1	7	3.125	0.4465	0.72506
1og5	CP2C9	6	2.671	0.4452	0.00772
1t67	HDAC8	6	2.619	0.4365	−0.2641
1s9j	MP2K1	9	3.921	0.4357	1.87334
2bu5	PDK2	6	2.602	0.4336	−0.6206
3bbt	ERBB4	6	2.559	0.4266	−0.4863
1qpe	LCK	6	2.554	0.4257	−0.5154
1mt6	SETD7	7	2.972	0.4246	1.25498
1w6j	ERG7	5	2.12	0.424	−1.7949
1hmt	FABPH	7	2.96	0.4228	0.21114
1fcy	RARG	8	3.38	0.4225	1.70098
2bk3	AOFB	7	2.953	0.4219	−0.046
1sa4	FNTA	7	2.952	0.4217	0.68966
1o1v	FABP6	7	2.94	0.42	0.258
1mzn	RXRA	7	2.939	0.4199	0.66477
1dkf	RARA	8	3.348	0.4185	1.5054
1svh	PRKACA	7	2.928	0.4183	1.01117
1p62	DCK	7	2.916	0.4166	0.87197
2w1g	AURKA	5	2.08	0.416	−1.6433
1nd5	PPAP	6	2.496	0.4159	−0.9438
2b7a	JAK2	7	2.888	0.4126	0.33259
1uwj	BRAF1	7	2.883	0.4119	0.34593
1tou	FABP4	6	2.471	0.4119	−0.3267
1y6b	VGFR2	7	2.874	0.4105	0.48752
2iko	RENI	7	2.867	0.4095	0.45273
1upw	NR1H2	6	2.444	0.4073	−1.0423
2fq9	CATS	5	2.035	0.4069	−1.1074
1nhz	GCR	8	3.238	0.4048	0.71596
1fe3	FABP7	7	2.804	0.4006	−0.2902
1nav	P10827	7	2.803	0.4004	−0.0991
1egc	ACADM	7	2.793	0.3989	0.90037
2ph6	BACE1	7	2.782	0.3974	0.42068
1l9n	TGM3	8	3.112	0.3889	0.43289
1q4n	AMY1	6	2.309	0.3849	−0.8531
1isj	BST1	7	2.648	0.3783	−0.135
1xap	RARB	9	3.388	0.3764	1.06752
2gpq	EIF4E	8	2.959	0.3699	1.48141
1i7b	DCAM	8	2.947	0.3684	1.12462
1jqe	HNMT	8	2.946	0.3683	0.07142
1gzu	NMNAT1	7	2.568	0.3668	−0.5435
2aeb	ARGI1	7	2.561	0.3658	−0.382
1hrk	FECH	8	2.925	0.3656	0.3439
2gqg	ABL1	8	2.923	0.3654	0.68279
1lv2	HNF4G	7	2.555	0.365	−0.8227
1qcf	HCK	7	2.542	0.3631	−0.8023
1kms	DYR	7	2.542	0.3631	−0.6051
1kqu	PLA2G2A	8	2.894	0.3617	0.02781
2i3i	BIRC7	8	2.883	0.3603	0.71932
1yv5	FPPS	8	2.872	0.359	0.01297
1nmy	KTHY	8	2.864	0.358	0.32451
1mlw	TPH1	7	2.505	0.3578	−0.832
1xbt	TK1	7	2.499	0.3571	−0.0525
1n46	THRB	7	2.498	0.3568	−0.5149
3dcu	NR1H4	8	2.852	0.3565	0.54104
1gbn	OAT	8	2.832	0.354	0.19086
1skx	NR1I2	10	3.519	0.3519	1.03581
1qvn	IL2	8	2.797	0.3496	0.02755
1p5j	SDS	7	2.432	0.3475	−1.1041
1itu	DPEP1	8	2.778	0.3473	−0.4048
1wb0	CHIT1	8	2.763	0.3453	0.35396
1fki	FKB1A	8	2.753	0.3442	−0.2358
1uym	HSP90AB1	8	2.732	0.3415	0.20683
1s0x	RORA	10	3.41	0.341	1.17973
1lt8	BHMT	8	2.714	0.3392	−0.027
1h9u	RXRB	10	3.359	0.3359	0.65611
1zpb	FA11	8	2.684	0.3355	0.04159
1x89	NGAL	7	2.297	0.3281	−1.7698
1g3m	ST1E1	7	2.269	0.3242	−1.4854
1jk7	PPP1CC	9	2.908	0.3231	0.27045
3cbs	CRABP2	9	2.899	0.3221	−0.2778
1tfg	TGFB2	9	2.897	0.3219	0.26176
1s19	VDR	8	2.553	0.3191	−0.5333
1y0s	PPARD	9	2.863	0.3181	0.37126
2oo8	TIE2	8	2.519	0.3149	−0.835
1xcw	AMYP	9	2.812	0.3124	0.49476
1gw6	LKHA4	9	2.794	0.3105	−0.0434
1hw9	HMDH	8	2.469	0.3086	−1.0548
2c6c	FOLH1	8	2.43	0.3038	−0.7386
1cm0	KAT2B	9	2.713	0.3015	−0.0951
1hfc	MMP1	8	2.41	0.3013	−1.0034
3ljr	GSTT2	11	3.313	0.3012	0.51526
2fgi	FGFR1	8	2.407	0.3008	−1.1558
1t46	KIT	9	2.659	0.2955	−0.3938
1o7a	HEXB	8	2.32	0.2901	−1.2444
1r6u	WARS	9	2.559	0.2844	−0.7534
1q91	NT5M	9	2.548	0.2831	−1.0567
2yxj	BCL2L1	9	2.53	0.2811	−0.6081
1xrj	UCK2	10	2.744	0.2744	−0.4852
1gre	GSR	9	2.457	0.273	−1.2507
1q5h	DUT	10	2.708	0.2708	−0.6111
1il0	HADH	11	2.946	0.2679	0.79201
1x0n	GRB2	9	2.336	0.2595	−1.6381
1liu	KPYR	9	2.335	0.2595	−1.4109
1njs	PUR2	11	2.833	0.2575	−0.1305
1nde	ESR2	9	2.302	0.2557	−1.4737
1dug	FIBG	11	2.792	0.2539	−0.4142
1g55	TRDMT1	10	2.509	0.2509	−1.0238
1bmq	CASP1	11	2.729	0.2481	−0.405
1kt8	BCAT2	11	2.723	0.2476	−0.4519
1p4m	RFK	12	2.952	0.246	0.03433
2auh	INSR	11	2.647	0.2406	−0.7274
1ln3	PCTP	11	2.403	0.2185	−1.3447
1r55	ADA33	10	2.175	0.2175	−1.8651
1l8j	EPCR	13	2.787	0.2144	−0.2622
1pbk	FKBP3	11	2.141	0.1946	−2.2826
1z6z	SPR	14	2.023	0.1445	−2.6542

**Figure 8:** GO and KEGG analyses. The top 20 signaling pathways of PTL in GO-Cellular Component analysis **(A)**. The top 20 signaling pathways of PTL in GO-Biological Process analysis **(A,B)**. The top 20 signaling pathways of PTL in GO-Molecular Function analysis **(C)**. The top 20 signaling pathways of PTL in KEGG pathways analysis **(D)**.

### The Combination of PTL and DDP Synergistically Inhibited the Activity of the PI3K/Akt Signaling Pathway in NSCLC Cells

Western blotting analysis demonstrated that both drug monotherapy and combination therapy increased the expression levels of Bax and cleaved Caspase-3, but decreased the expression levels of p-PI3K, p-Akt, Caspase-3, and Bcl-2, with total expression levels of Akt, PI3K, and glyceraldehyde 3-phosphate dehydrogenase remaining unchanged. Importantly, the efficacy of drug combination treatment was more significant than the single drug treatments (PTL + DDP vs. PTL, *p* < 0.01; PTL + DDP vs. DDP, *p* < 0.01). Moreover, the inhibitory effect of PTL + DDP combined treatment on the signaling pathway was partially restored by a PI3K activator (740 Y-P), as shown in Figure 9 (*p* < 0.01 for p-PI3K, p-Akt, Caspase-3, Bcl-2, Bax, and cleaved Caspase-3 between 740 Y-P + PTL + DDP and PTL+ DDP groups).

**Figure 9:** Suppressive effect of PTL, DDP, and the combination on the PI3K/AKT signaling pathway in A549 cells. Protein expression levels of p-PI3K, PI3K, p-Akt, Akt, Caspase-3, cleaved Caspase-3, Bcl-2, Bax, and GAPDH in A549 cells treated with 30 μM PTL, 0.75 μM DDP alone, and 0.2 μM DDP and 10 μM PTL in combination with or without 30 μM 740 Y-P for 48 h **(A)**. Histograms depicting the relative gray value of the related proteins measured using ImageJ **(B–E)**. All data are shown as the mean ± SD of three independent experiments. *P < 0.05, **P < 0.01 or ***P < 0.001 vs. the control group.

## Discussion

In the process of tumor chemotherapy, one of the toughest problems is that cancer cells develop resistance to chemotherapy drugs. Despite the fact that cisplatin-based chemotherapy is the first-line therapy for NSCLC, the occurrence of acquired resistance to cisplatin still presents a great challenge (Dasari and Tchounwou, 2014; Rossi and Di Maio, 2016). The development of cisplatin resistance is a key issue in the failure of NSCLC therapy, and can lead to cancer palindromia and metastasis.

Artemisinin (qinghaosu) and arsenic oxide (III) (As_2_O_3_) have achieved remarkable success in clinical practice, and have attracted the attention of many researchers to natural extracts. Considering their safety, long-term use, and ability to target various pathways, there has been great interest in re-understanding the molecular mechanisms of their activities. In the clinical practice, many traditional Chinese medicines have shown synergistic effects in chemotherapy.

In recent years, PTL has shown the ability to comprehensively prevent tumor progression, such as the prevention of NSCLC through the induction of apoptosis. Although PTL has been reported to have anti-tumor ability, the mechanism by which it inhibits tumorigenesis remains unclear. Therefore, to fully explain its biological activity on different types of cancer, including NSCLC, will require further research. According to modern pharmacological research, the combined application of two drugs could inhibit the growth, proliferation, migration, and invasion of a variety of tumor cells, as well as induce tumor cell apoptosis and inhibit the effect of tumor-promoting substances on potential tumor cells. In this study, we found that the combined use of PTL and DDP had a synergistic effect on NSCLC. This can be considered as a new adjuvant treatment strategy for NSCLC.

Some recent studies have also provided evidence that PTL could act against many varieties of cancers, such as NSCLC (Talib and Al Kury, 2018) and breast cancer (Araujo et al., 2019; Berdan et al., 2019). Nevertheless, there is a lack of evidence at both cellular level and in animal models to show the effect of PTL and DDP combination on the development of NSCLC. This study revealed that PTL combined with DDP had an inhibitory effect on the growth and metastasis of NSCLC and the PI3K/Akt pathway, providing a potential basis for the promising strategy of PTL and DDP combination for the treatment of NSCLC.

According to the IC_50_ values analyzed using CCK8 assay, we proved that PTL and DDP could inhibit the proliferation of A549, PC9, and H1299 cells in a dose-dependent and time-dependent manner. In comparison with PTL, DDP had a stronger inhibitory effect on the tested cell line when treated as a single agent. The combination of drugs exerted a synergistic inhibitory effect on A549, PC9, and H1299 cells. Based on the above results, we proposed the hypothesis that PTL may increase the sensitivity of NSCLC to DDP.

Furthermore, PTL can not only inhibit hypoxia-inducible factor-1α signaling transduction in colorectal cancer, but could also inhibit hypoxia induced epithelial-mesenchymal transition (Kim et al., 2017). As suggested by our findings, the combination of PTL and DDP could synergistically suppress the migration and invasion ability of A549 and PC9 cells.

In addition, this study analyzed the mechanism of the synergistic effect of PTL and DDP on cell cycle distribution in A549 and PC9 cells using FCM. The results indicated that PTL, DDP, and combined treatment caused S and G2 phase arrest in A549 and PC9 cells. Tang found that PTL treatment inhibited survivin, arrested cancer cells at G2/M phases, and triggered cell death in human malignant glioblastoma cells (Tang et al., 2015). However, there is still a controversy in terms of the effect of PTL on cell cycle distribution. One study using human uveal melanoma cells discovered diverse outcomes that PTL exerted growth-inhibiting and apoptosis-inducing effects in UM cells by blocking G1 phase and regulating the mitochondrial pathway (Che et al., 2019). These findings showed that PTL may be conducive to cell cycle arrest at G1 phase in human uveal melanoma cells, while PTL might lead to G_2_/M phase cell cycle arrest in human malignant glioblastoma cells, both of which necessitate further discussion.

Numerous studies have showed that PTL suppresses tumor-promoting effects of nicotine in lung cancer through inducing p53-dependent apoptosis (Talib and Al Kury, 2018), adjusts mitochondrial autophagy induced by oxidative stress, and plays an inhibitory role in the apoptosis of C2C12 myoblasts *via* the p53 signaling pathway (Ren et al., 2019). Our study also revealed that, in A549 and PC9 cells, the same results were achieved with both PTL and DDP, and that apoptosis rates could be improved remarkably with their combined application rather than with monotherapy. Overall, these results indicated that apoptosis could be synergistically promoted by a combination treatment of PTL and DDP.

Moreover, PTL was discovered to induce intrinsic apoptosis in thyroid carcinoma cells both *in vivo* and *in vitro* by Li C's team (Yang et al., 2019). Our research showed that both PTL and DDP could suppress the growth of NSCLC xenograft tumors, and that more significant effects were observed with their combination *in vivo*. As a result, our results showed that the anti-tumor effect of DDP could be effectively enhanced by PTL *in vivo*. Because of lack of funds, the number of animals we were able to experiment on was limited. Therefore, we did not have different (i.e., less frequent) Schedules of Administration.

Next, the relevant information of the first 300 potential protein targets of PTL was acquired utilizing PharmMapper (Wang et al., 2017). Due to the KEGG pathway analysis, we realized that PTL, in line with recent studies, may chiefly affect the PI3K/Akt signaling pathway (Jeyamohan et al., 2016; Yang et al., 2019). Likewise, according to numerous current investigations, the chemosensitivity of NSCLC cells to DDP could be increased through the inactivation of the PI3K/Akt pathway (Chen et al., 2017; Shi et al., 2017; Gong et al., 2018; Liu et al., 2018; Xia et al., 2018; Zhao et al., 2018). We therefore speculated that PTL may improve the anti-tumor ability of DDP in NSCLC by obstructing the PI3K/Akt pathway.

There are various cellular processes such as survival, proliferation, growth, metabolism, angiogenesis, and metastasis that can be regulated by the hyperactivated or altered PI3K/Akt/mammalian target in the rapamycin (mTOR) signaling pathway in many cancer types (Katso et al., 2001; Engelman et al., 2006; Martini et al., 2014). The development of cancer resistance to anticancer therapies is closely related to the activation of the PI3K/AKT/mTOR pathway in several tumor types (Martini et al., 2014). PI3Ks are a group of lipid kinases related to the plasma membrane and are composed of three subunits, the p85 regulatory subunit, the p55 regulatory subunit, and the p110 catalytic subunit (Donahue et al., 2012). Based on their diverse structures and particular substrates, PI3Ks are classified into three classes: I, II, and III (Hennessy et al., 2005; Engelman et al., 2006; Martini et al., 2014; Asati et al., 2016). Over the past few decades, the PI3K pathway has been thought to be deregulated in multiple human cancers, including NSCLC (Dillon et al., 2007). The PI3K pathway is inactivated by various mechanisms, including the tumor suppressor PTEN, variation or expansion of PI3K, and activation of the upstream tyrosine kinase growth factor receptor or oncogene of PI3K (Stemke-Hale et al., 2008). It was found that overactivity of the PI3K signaling pathway was significantly correlated with the progression of human tumors, increased tumor microvascular density, chemotaxis, and enhanced invasion of cancer cells. Therefore, the PI3K signaling pathway has been considered one of the main targets for cancer therapy (Hennessy et al., 2005; Dillon et al., 2007). Great efforts have been made to develop drugs targeting the PI3K signaling pathway, with many presently being evaluated in clinical tests (Aziz et al., 2009). The suppression of PI3K signaling is a promising and valid means for the treatment of NSCLC.

Through Western blotting, we found that drug treatment resulted in a significant increase in the expression levels of cleaved Caspase-3 and Bax, but the expression levels of Bcl-2, Caspase-3, p-Akt and p-PI3K proteins were lower, and total Akt and PI3K protein expression remained unchanged. In comparison with single-agent therapy, the combination treatment exhibited a greater effect. Therefore, we proposed a hypothesis that the drug-induced pro-apoptotic process may be related to the downregulation of the PI3K/Akt signaling pathway. In keeping with numerous other research studies, our findings suggested that based on the upregulation of Bax and cleaved Caspase-3, the mitochondrial apoptotic pathway was related to PTL-induced A549 cell death. Unfortunately, we have not validated studies from other perspectives, such as whether AKT inhibition reproduces the effect of PTL on DDP sensitivity, and there remains a lack of further study of the upstream mechanisms of AKT.

The above studies showed that inhibiting the PI3K/Akt signaling cascade could be considered an effective strategy for NSCLC therapy. Drugs targeting the apoptosis pathway (such as PTL) may also serve as an effective strategy for NSCLC therapy, and might play vital roles in minimizing adverse reactions, maximizing clinical efficacy, and helping to increase the quality of life for patients.

According to the results of our research, PTL combined with DDP could synergistically suppress NSCLC cells through the downregulation of the PI3K/Akt signaling pathway. In combination therapy, PTL was able to increase the sensitivity of NSCLC cells to DDP, allowing for its reduced dose, thereby potentially decreasing its side effects. This discovery provides the basis for PTL as a new option for combination therapy in the treatment of NSCLC.

In summary, our study showed that PTL could strengthen the pro-apoptotic effect of DDP on NSCLC cells through arresting cells at S and G2/M phases, thus functioning as an inducer of apoptosis. In the xenograft models, PTL and DDP combination demonstrated distinct anti-cancer activity and reduced tumor volumes and weights. Therefore, PTL has potential as a synergistic drug in combination with DDP to prevent NSCLC.

## Data Availability Statement

The raw data supporting the conclusions of this article will be made available by the authors, without undue reservation.

## Ethics Statement

The animal study was reviewed and approved by Institutional Animal Care and Use Committee of Sun Yat-sen University.

## Author Contributions

W-HC, J-FZ, Z-RH, and S-QN designed the research. L-MW, X-ZL, BK, LS, and YZ performed the experiments. L-MW, X-ZL, BK, LS, and YZ performed the data analysis. W-HC, J-FZ, Z-RH, and S-QN contributed to the guidance of the experiments. L-MW, X-ZL, and YZ wrote the manuscript. W-HC and J-FZ edited and revised the manuscript. All authors authorized the final version of the manuscript.

## Conflict of Interest

The authors declare that the research was conducted in the absence of any commercial or financial relationships that could be construed as a potential conflict of interest.

## Abbreviations

2D: two dimensional
CCK8: Cell Counting Kit-8
CI: combination index
CID: compound ID
cisplatin: DDP
ECL: electrochemiluminescence system
Fa: fraction affected
FCM: flow cytometry
HRP: horseradish peroxidase
NSCLC: non-small-cell lung cancer
PI: propidium iodide
PI3K: phosphatidylinositol 3-kinase
PTL: parthenolide
PVDF: polyvinylidenedifluoride
TCM: Traditional Chinese medicine.
